# Elucidating the life cycle of opossum parasites: DNA sequences reveal the involvement of planorbid snails as intermediate hosts of *Rhopalias* spp. (Trematoda: Echinostomatidae) in Brazil

**DOI:** 10.1371/journal.pone.0279268

**Published:** 2023-03-03

**Authors:** Danimar López-Hernández, Marisa Caixeta Valadão, Alan Lane de Melo, Vasyl V. Tkach, Hudson Alves Pinto

**Affiliations:** 1 Departamento de Parasitologia, Laboratório de Biologia de Trematoda, Instituto de Ciências Biológicas, Universidade Federal de Minas Gerais, Belo Horizonte, Minas Gerais, Brazil; 2 Department of Biology, University of North Dakota Grand Forks, Grand Forks, ND, United States of America; Nanjing Agricultural University, CHINA

## Abstract

Echinostomatid digeneans belonging to the genus *Rhopalias* are intestinal trematodes found mainly in opossums in the New World. The genus comprises seven species, but their life cycles and intermediate hosts have been unknown until now. During our long-term study carried out in freshwater habitats within the state of Minas Gerais, Southeast Brazil, echinostomatid cercariae lacking collar spines were found in planorbid snails *Biomphalaria glabrata*, *Biomphalaria straminea*, *Drepanotrema lucidum* and *Gundlachia ticaga* in six different batches of snail samples collected between 2010 and 2019. Morphologically, the larvae reported herein are morphologically consistent with each other and characterized by the presence of 2–3 large ovoid or spherical corpuscles in each main duct of the excretory system, resembling to *Cercaria macrogranulosa* previously described from the same region of Brazil. Partial sequences of the ITS (ITS1-5.8S-ITS2) region and 28S gene of the nuclear ribosomal RNA operon, and partial sequences of mitochondrial *nad*1 and *cox*1 genes were obtained and compared with the data available for members of the family Echinostomatidae. Nuclear markers indicate that all samples of cercariae evaluated in the present study can be assigned to *Rhopalias*, but distinct from North American isolates of *Rhopalias macracanthus*, *Rhopalias coronatus* and *Rhopalias oochi* (divergence 0.2–1.2% in 28S and 0.8–4.7% in ITS). The lack of differences verified in both 28S and ITS in 5 out 6 studied samples suggested that they belong to the same species. However, *nad*1 sequences revealed that our cercariae correspond to three distinct species of *Rhopalias* (interspecific divergence: 7.7–9.9%), named here as *Rhopalias* sp. 1, found in *B*. *straminea* and *G*. *ticaga*, *Rhopalias* sp. 2 found in *B*. *glabrata* and *D*. *lucidum*, and *Rhopalias* sp. 3 also found in *D*. *lucidum*. They also differ by 10.8–17.2% from a North American isolate of *R*. *macracanthus* sequenced in this study. The *cox*1 sequences obtained for *Rhopalias* sp. 1 and *Rhopalia*s sp. 2 (but not *Rhopalia*s sp. 3) reveal that they are distinct from North American isolates of *R*. *macracanthus* (genetic divergence 16.3–16.5% and 15.6–15.7%, respectively), *R*. *coronatus* (9.2–9.3% and 9.3–9.5%) and *Rhopalias oochi* (9.0% and 9.5–10.1%). Encysted metacercariae with general morphology similar to that of the body of cercariae were found in tadpoles of *Rhinella* sp. from the same stream where snails harbored *Rhopalias* sp. 2, suggesting that the amphibians could act as second intermediate hosts of species of *Rhopalias*. Data obtained provide the first insights into the life cycle of this unusual echinostomatid genus.

## Introduction

Echinostomatid digeneans belonging to the genus *Rhopalias* Stiles and Hassall, 1898 are intestinal flukes found mainly in didelphid opossums (occasionally reported in bats, rodents, and birds) in the Americas [1–4]. Species of the genus *Rhopalias* are unique among the echinostomatoideans due to the presence of two eversible proboscises armed with spines situated symmetrically on either side of the oral sucker [1, 3–5]. In the past, *Rhopalias* was included in the family Rhopaliidae Looss, 1899, as the type and only genus. However, this family was recently synonymized with the Echinostomatidae Looss, 1899 by Tkach et al. [6] based on molecular phylogenetic analyses.

Currently, seven species of *Rhopalias* are considered valid [4, 5]. The type-species of the genus, *Rhopalias coronatus* (Rudolphi, 1819), was originally described from marsupials in Brazil [3, 7, 8]. Although reports of species of *Rhopalias* in definitive hosts are not uncommon, the intermediate hosts and life cycle of these trematodes remain unknown. As with most digenean groups, this deficiency in understanding basic life-history can partially be explained by the methodological difficulties associated with classical experimental approach used to study helminth life cycles [9]. Probably the apparent specificity to marsupials as definitive hosts makes experimental studies involving *Rhopalias* more complicated compared with other echinostomes, given the difficulties of maintaining such types of wild vertebrates under laboratory conditions.

The introduction of DNA sequencing has accelerated the elucidation of life cycles of trematodes [9, 10], including representative species of the superfamily Echinostomatoidea Looss, 1902 [11–17]. However, no sequence data from *Rhopalias* spp. were available. Recently, sequence data for adult stages of three species of *Rhopalias* in North America have been made available [5, 6, 18], enabling molecular matching with other life cycle stages.

Herein, we present the results of morphological and molecular studies of echinostomatid larvae found in planorbid snails from Brazil that enabled us to identify for the first time cercariae of *Rhopalias* spp. Moreover, we obtained evidence of the probable involvement of anurans as the second intermediate hosts of these digeneans. We also examined phylogenetic relationships within *Rhopalias* using new and previously published sequence data.

## Materials and methods

### Sample collection

The present study is part of long-term malacological and helminthological surveys carried out in freshwater habitats across the state of Minas Gerais, southeast Brazil, between 2010 and 2019. Snails were collected with a dip net and transported to the laboratory, where they were individually placed in polystyrene plates and exposed to light for about 2 hrs. After this period, the water was examined with a stereomicroscope to detect the shedding of cercariae. The plates were examined again the next day, before and after a new period of photostimulation. Some of the infected snails were crushed between glass plates and examined for the presence of rediae. The taxonomic identifications of the snail species were based on morphological traits (shell and internal anatomy) [19–22]. The species, localities and date of collection of the snails infected with larval trematodes used for this study are provided in Table 1.

**Table 1:** Data on the studied cercarial samples collected from planorbid snails in the state of Minas Gerais, Brazil.

HOST	LOCALITY	GCS	DATE	GENBANK ACCESSION NUMBERS			
				28S	ITS	*cox*1	*nad*1
*Biomphalaria straminea*	Belo Horizonte	19°50’18"S,	06-06-2012	OP972553	OP972548	OP971532	OP980993
		43°59’40"W					
*Gundlachia ticaga*	Belo Horizonte	19°50′17"S,	05-11-2017	—	OP972549	—	OP980994
		43°57′32"W					
*Biomphalaria glabrata*	Januária	15°29’41"S,	06-07-2010	OP972554	—	OP971533	OP980995
		45°08’59"W					
*Biomphalaria glabrata*	Januária	15°29’41"S,	08-29-2019	OP972555	OP972550	—	OP980996
		45°08’59"W					
*Drepanotrema lucidum*	Patos de Minas	18°42’33"S,	07-19-2019	OP972556	OP972551	OP971534	OP980997
		46°35’04"W					
*Drepanotrema lucidum*	Dores do Indaiá	19°29’41"S,	12-25-2013	OP972557	OP972552	—	OP980998
		45°36’46”W					

### Molecular study

Aiming to identify and distinguish the species found, as well as to place these within an echinostomatid phylogeny, six samples of echinostome cercariae lacking collar spines were subjected to molecular analysis. Each sample evaluated corresponds to larvae shed by a same infected snail. About 30 ethanol-fixed cercariae from each sample were used for molecular study. DNA was extracted from the pooled cercariae using the QIAamp DNA micro kit (Qiagen Ltd., Crawley, United Kingdom), according to the manufacturer’s instructions. The concentration of the extracted DNA was determined using a NanoDrop Lite spectrophotometer (Thermo Fisher Scientific, Wilmington, USA). Attempts were made to amplify partial fragments of 28S (primers digl2/1500R; [23]) and internal transcribed spacer region (primers BD1/BD2; [24]) regions of the nuclear ribosomal operon, and of mitochondrial genes *nad*1 (NDJ11 and NDJ2a; [25] or JB11 and JB12; [26]) and *cox*1 (Dice-1 and Dice-11 [27]; Dice-1 and BarCox-R [5]). DNA amplifications were performed by polymerase chain reaction (PCR) following the PCR conditions described by the authors listed above. PCR reactions were done using Platinum™ Hot Start PCR Master Mix (2X) (Thermo Fisher Scientific) according to the manufacturer’s instructions, 10 μM of each primer and about 50 ng of DNA. Positive PCR products were purified using polyethylene glycol 8000 (20%) (Promega, Madison, WI), according to [28].

The obtained amplicons were sequenced in both directions using the BigDye Terminator Cycle Sequencing Ready Reaction Kit (Applied Biosystems, Inc., Foster City, CA) and the same primers as used in PCR reactions. Sequencing reactions were cleaned using a BigDye Sequencing Clean Up Kit (MCLAB, California, USA.) and run on an ABI 3130 automated capillary sequencer (Thermo Fisher Scientific, Waltham, Massachusetts, USA). An adult specimen of *Rhopalias macracanthus* Chandler, 1932 previously collected from a specimen of the Virginia opossum, *Didelphis virginiana* Kerr, 1792 from North Carolina, USA, by one of the authors (VVT) was sequenced using the same primers and PCR conditions as described above.

The obtained sequences were visualized and assembled in ChromasPro (Technelysium Pty Ltd, Australia). The resulting contiguous sequences were aligned with sequences of selected echinostomatid taxa available in GenBank using MEGA X [29]. The alignments were each trimmed to the shortest sequence. Unreliable positions (ambiguous homology) in the alignments were identified and excluded using the Gblocks web server (http://phylogeny.lirmm.fr/) [30]. Six new 28S sequences (5 for the cercariae from Brazil and 1 for adult from USA) were obtained (1052–1186 bp) and final alignment consisted of 31 sequences and was 1077 bp long (4 ambiguous positions excluded). For ITS, we analyzed the whole fragment (ITS1-5.8S-ITS2) as well as the ITS2, because the whole region is not available for several taxa of the Echinostomatoidea. For this molecular marker, five new ITS sequences (994 bp) were obtained and a dataset containing 19 sequences was evaluated (954 bp long; 12 ambiguous positions removed). In the case of ITS-2, the analysis was based on 17 sequences and a trimmed alignment of 378 bp (7 ambiguous positions excluded). We obtained *nad*1 sequences (332–413) bp from the six samples of cercariae and the final dataset consisted of 42 sequences and 398 bp. For *cox*1, three sequences were generated (612 bp, 643bp and 675bp), and the final dataset consisted of 33 sequences with a trimmed alignment of 612 bp. Phylogenetic reconstructions were performed by Bayesian inference (BI) and maximum likelihood (ML) methods using the programs MrBayes v.3.2.6 [31] and MEGA X [29], respectively. The best nucleotide substitution models were determined according to the Bayesian Information Criterion in MEGA X. The best fitting models were: GTR+G+I for 28S data; K2+G for ITS and ITS2 data; GTR+G+I for *nad*1, and HKY+G+I for *cox*1. The selection of outgroups was based on the phylogeny of the Echinostomatoidea by Tkach et al. [6]. The ML trees were generated via MEGA X and the nodal support was estimated using the bootstrap method with 1,000 pseudoreplicates. BI analyzes were performed using Markov chain Monte Carlo (MCMC) in two simultaneous runs of four chains for 1,000,000 generations and sampling every 100 generations. The first 25% of the sampled BI trees were discarded as ’burn-in’. Phylogenetic trees and data files were visualized in FigTree version 1.4.3 [32]. The new sequences obtained in this work were deposited in GenBank (Table 1).

### Morphological study

Cercariae that emerged from naturally infected snails were stained with vital dyes (aqueous solution of 0.05% neutral red or Nile blue sulfate), wet mounted and examined under a light microscope. Cercariae for the morphometric study were killed in water at 70°C and fixed in 10% formalin. Subsequently, they were temporarily mounted between slide and coverslip and measured using an ocular micrometer. Some of the fixed cercariae were stained in alum acetocarmine, dehydrated in graded ethanol series, cleared in beechwood creosote, and mounted on permanent slides. Rediae were studied alive on temporary wet mounts. Photographs were taken with a Leica ICC50 HD digital camera coupled to a light microscope. Morphological characterization and preliminary identification of the cercariae were based on descriptions of digenean larvae reported in South America [33–36]. All measurements in morphological descriptions are shown in micrometers as mean ± standard deviation and range in parentheses.

### Experimental infection

In order to obtain metacercariae experimentally, we attempted to infect laboratory-reared snails [*Biomphalaria glabrata* (Say, 1818)] and fish (*Poecilia reticulata* Peters, 1859). These species were used as experimental hosts due to their availability in the laboratory and previous knowledge on the involvement of snails and fish as second intermediate hosts of echinostomes. The behavior of cercariae in the presence of these potential hosts was observed under a stereomicroscope. After 24hs of exposure to cercariae, the snails and fish were necropsied. We also searched for metacercariae in samples of insects, fishes, snails, and tadpoles collected in the same water bodies where snails were found infected.

Metacercariae found in tadpoles collected in the stream where snails were found infected were used for an experimental infection study. We suspected they could be of the same species based on the number of excretory corpuscles. Aiming to obtain adult parasites for taxonomic identification, a sub-sample of 50 metacercariae was orally administered to one specimen of a dexamethasone-immunosuppressed (50 mg/kg) male Swiss mouse. The infected mouse was maintained on a 12/12h light–dark cycle and allowed access to food and water ad libitum. Coproparasitological examinations by the sedimentation technique were conducted daily, starting from seven days post-infection. The mouse was euthanized via barbituric overdose (sodium pentobarbital, injected intraperitoneally) and necropsied for the search of adult parasites 14 days post-infection.

### Ethics statement

The snails were collected under authorization by the Brazilian Institute of Environment and Renewable Natural Resources (IBAMA) (SISBIO 52870–1). Experimental studies were approved by the local Ethics Committee on Animal Use of the Universidade Federal de Minas Gerais (CEUA -UFMG, protocol 20/2016).

## Results

### Molecular study

For this study, six samples of morphologically similar unspined echinostome cercariae were used in the molecular study (Table 1). Analyses of novel molecular data from these infections are consistent with the presence of three species, and suggest that all three represent species of the genus *Rhopalias*, referred to here as *Rhopalias* sp. 1–3. Our phylogenetic analyses based on the partial ITS and 28S revealed that sequences of all larval samples obtained in this study appeared in well-supported clades with sequences of the two isolates of adult *R*. *coronatus* and *R*. *macracanthus* from marsupials (Fig 1). This finding provides clear evidence that the cercariae found in this study in planorbid snails from Brazil belong to the genus *Rhopalias*. Most of new 28S sequences generated from cercariae evaluated in this study were identical each other, except for the cercariae found in *D*. *lucidum* from Dores do Indaiá, which differed in 1%. The genetic divergence found for this same molecular marker between the Brazilian cercariae and previously and new adult-based sequences of *Rhopalias* spp. ranged from 0.23 to 1.34%. The intergeneric differences between species of *Rhopalias* and those of the sister genera *Ribeiroia* [*Ribeiroia ondatrae* (Price, 1931) from USA, *Ribeiroia* sp. 2 and *Ribeiroia* sp. 3 from Kenya] and *Cathaemasia* [*Cathaemasia hians* (Rudolphi, 1809) from Czech Republic] were 4.1–4.9% and 2.7–3.1%, respectively.

**Fig 1:** Phylogenetic relationships between *Rhopalias* spp. found in planorbids from Brazil and members of the family Echinostomatidae inferred from partial 28S sequence data (1077 bp). The trees were generated by Bayesian Inference (BI) and Maximum Likelihood (ML) methods. New sequences from the present study are in bold. Scale bar represents the number of nucleotide substitutions per site.

Similar to 28S data, the phylogenetic analyses based on ITS also revealed a clade formed by our samples and North American isolates of *R*. *macracanthus*, *Rhopalias oochi* López-Caballero, Mata-López, Pérez-Ponce de León, 2019 and *R*. *coronatus* (Fig 2A). The genetic divergence between the Brazilian samples was 0–1.2%; they differed from North American isolates of *R*. *macracanthus*, *R*. *oochi* and *R*. *coronatus* by 0.6–4.7%. Only ITS-2 data were available for comparison with the species of the sister genera *Ribeiroia* and *Cathaemasia*. also revealed that the species of both genera form a clade with *Rhopalias* spp. (Fig 2B), although in this tree the clade of *Ribeiroia* spp. was nested among lineages of *Rhopalias*. The intergeneric differences between *Rhopalias* spp. and *Ribeiroia* spp. and *C*. *hians* were 7.7–8.6% and 5.6–7.2%, respectively.

**Fig 2:** Phylogenetic relationships between *Rhopalias* spp. found in planorbids from Brazil and members of the family Echinostomatidae inferred from (A) ITS1-5.8S-ITS-2 (954 bp) and (B) ITS2 (378 bp) sequence data. The trees were generated by Bayesian Inference (BI) and Maximum Likelihood (ML) methods. New sequences from the present study are in bold. Scale bar represents the number of nucleotide substitutions per site.

The tree resulting from molecular phylogenetic analyses based on *nad*1 sequences showed 6 cercarial samples sequenced in this study, in three different clades, interpreted here as representing three different species of *Rhopalias* (Fig 3A). The pairwise comparison between the *nad*1 sequences obtained for the six samples evaluated in this study is presented in Table 2. Sequences from cercariae found in *Biomphalaria straminea* (Dunker, 1848) and *Gundlachia ticaga* (Marcus & Marcus, 1962) collected in two urban lakes from Belo Horizonte, were identical and named herein *Rhopalias* sp. 1. Cercariae found in *B*. *glabrata* from Januária and *Drepanotrema lucidum* (Pfeiffer, 1839) from Patos de Minas differ by merely 2.1–2.4%, suggesting these parasites belong to the same species, named here *Rhopalias* sp. 2. It differs from *Rhopalias* sp. 1 in 7.7–8.4%. The cercariae found in *D*. *lucidum* from Dores do Indaiá differs by 9.9% and 9.8–9.9% from *Rhopalias* sp. 1 and *Rhopalias* sp. 2, suggesting it is a distinct species, *Rhopalias* sp. 3. Moreover, *nad*1 sequence data for samples of these three species formed a clade, and samples of each species grouped in the respective subclades. The *nad*1 sequence of the North American isolate that morphologically corresponds to *R*. *macracanthus*, showed 10.8–17.2% divergence from 3 *Rhopalias* spp. from Brazil collected in this study as cercariae. Moreover, in the phylogenetic analyses based on *nad*1, this isolate of *R*. *macracanthus* grouped in a distinct subclade with *Rhopalias* sp. 3, but the nodal support was low. Genetic divergences between *Rhopalias* spp. and selected species from 6 genera of the Echinostomatidae that were included in the analyses ranged from 20.7 to 36.1%.

**Fig 3:** Phylogenetic relationships between *Rhopalias* spp. found in planorbids from Brazil and members of the family Echinostomatidae inferred from (A) *nad*1 (397 bp) and (B) *cox*1 (612 bp) sequence data. The trees were generated by Bayesian Inference (BI) and Maximum Likelihood (ML) methods. New sequences from the present study are in bold. Scale bar represents the number of nucleotide substitutions per site.

**Table 2:** Pairwise distances (uncorrected p-distance) based on *nad*1 sequences obtained from cercariae of *Rhopalias* spp. found in planorbid snails from Brazil.

	#1	#2	#3	#4	#5
*Rhopalias* sp. 1 –*Biomphalaria straminea*					
*Rhopalias* sp. 1 –*Gundlachia ticaga*	0%				
*Rhopalias* sp. 2 –*Biomphalaria glabrata*	8.28%	8.88%			
*Rhopalias* sp. 2 –*Biomphalaria glabrata*	7.67%	8.31%	1.83%		
*Rhopalias* sp. 2 –*Drepanotrema lucidum*	8.43%	8.43%	2.41%	2.11%	
*Rhopalias* sp. 3 –*Drepanotrema lucidum*	9.94%	9.94%	9.76%	9.94%	9.94%

Data obtained for *cox*1 gene confirmed the presence of two species in the samples evaluated for this marker. *Rhopalias* sp. 1 differs by 7.3–7.9% from *Rhopalias* sp. 2. The isolates of this last species from Patos de Minas and Januária differed 1.31%. The two sequenced Brazilian species differ by 9.2–9.5% from *R*. *coronatus* and 9.0%–10.1% from *R*. *oochi*. In the *cox*1 tree, the Mexican isolates of *R*. *coronatus* and *R*. *oochi* appeared in a separate sub-clade from Brazilian *Rhopalias* sp. 1 and *Rhopalias* sp. 2 (Fig 3B). The two Brazilian isolates differ by 15.2–16.5% from a Mexican isolate of *R*. *macracanthus* and by 12–13.1% from the North American sample of the same species sequenced in this study. Notably, the divergence between the two isolates of *R*. *macracanthus* from Mexico and the USA was very high (15%) clearly demonstrating that these isolates are not conspecific. The levels of sequence divergence between *Rhopalias* spp. and other species of echinostomatids included in the *cox*1 analyses were high at 21.8–25.1%.

### Morphological and experimental studies

No apparent morphological differences were found between the cercariae of the three species of *Rhopalias* found in different species of planorbids from different localities in the state of Minas Gerais, Brazil. Measurements of cercariae from four of the collected samples are shown in Table 3, along with the data available for similar larvae reported by different authors in South America.

**Table 3:** Morphometric data of larval stages of *Rhopalias* spp. examined in this study, and other unspined echinostome cercariae described in South America by different authors.

		*Rhopalias* sp. 1	*Rhopalias* sp. 2	*Rhopalias* sp. 2	*Rhopalias* sp. 3	*Cercaria macrogranulosa*		*Cercaria echinostoma 2*	*Cercaria guaibensis 8*
**Reference**		Present study				Ruiz, 1952 [33]	Ostrowski de Núñez et al., 1990 [36]	Veitenheimer- Mendes, 1982 [34]	Veitenheimer- Mendes et al., 1995 [35]
**Locality**		Belo Horizonte, MG, Brazil	Patos de Minas, MG, Brazil	Januária, MG, Brazil	Dores do Indaiá, MG, Brazil	Belo Horizonte, MG, Brazil	Parana River Basin, Argentina	Camaquã, RS Brazil	Porto Alegre, RS Brazil
**Host**		*Biomphalaria straminea*	*Drepanotrema lucidum*	*Biomphalaria glabrata*	*Drepanotrema lucidum*	*Biomphalaria glabrata*	*Drepanotrema depressissimum*	*Biomphalaria peregrina*	*Drepanotrema depressissimum*
Body	L	248±12 (232–280)	220±30 (149–269)	217±15 (248–177)	211±14 (186–229)	215–283	242±11 (218–260)	222–249	360
	W	132±8 (123–157)	118±27 (78–199)	133±8 (149–121)	124±14 (107–150)	91	96±8 (84–105)	111–127	–
Tail	L	449±14 (423–478)	438±24 (383–468)	411±15 (432–355)	368±18 (350–400)	340–493	436±19 (420–470)	360–407	420
	W	52±4 (47–62)	41±6 (36–57)	39±4 (43–28)	50±8 (36–57)	–	46±4 (42–50)	37–55	–
Oral	L	43±1(42–45)	38±3 (32–45)	42±3 (45–36)	45±4 (39–53)	40–47	38±3 (31–42)	34–41	45
sucker	W	43±1 (42–45)	37±3 (32–53)	42±3 (46–36)	48±4 (44–53)	–	39±3 (31–42)		–
Ventral	L	50±3 (45–57)	47±6 (32–59)	46±5 (63–36)	54±11 (35–69)	54–70	57±5 (48–63)	48–67	55
sucker	W	56±3 (52–58)	55±7 (35–72)	63±4 (71–54)	58±7 (51–70)	–	60±5 (52–69)	–	–
Pharynx	L	21±2 (18–25)	18±4 (14–21)	25±5(36–18)	21±7 (12–26)	–	20±7 (21–25)	–	–
	W	17±1 (15–18)	15±2 (13–18)	17±6 (36–11)	20±7 (12–23)	–	18±3 (10–23)	–	–

All measurements are in micrometers; mean values are followed by the standard deviation and range in parentheses. Abbreviations: L: length; W: width.

We did not observe any change in the behavior of cercariae of *Rhopalias* sp. 1 placed in contact with laboratory-reared *B*. *glabrata*. No metacercariae were found in these invertebrates 24 hrs. after exposure, indicating that at least this snail species was not a suitable second intermediate host for this digenean. On the other hand, encysted metacercariae and free tails were observed in the wells containing *P*. *reticulata* thirty minutes after the exposure to cercariae. Moreover, a few cysts were found in the oral cavity of the fish necropsied 24 hrs after infection. Specimens of experimentally infected fish examined after this period had a few dead metacercariae in the oral cavity. However, beyond the fact that the contact with these fish induced encystment, our data suggest that *P*. *reticulata* is likely not a suitable second intermediate host for species of *Rhopalias*. On the other hand, we found metacercariae morphologically reminiscent of *Rhopalias* cercariae in the kidneys of *Rhinella* sp. tadpoles caught in the same stream where *Rhopalias* sp. 2 from Januária were collected. No adult worm was found in the mouse experimentally orally inoculated with metacercariae obtained from these naturally infected tadpoles.

### Taxonomic summary

Class Trematoda Rudolphi, 1808
Superfamily Echinostomatoidea Looss, 1899
Family Echinostomatidae Looss, 1899
Genus *Rhopalias* Stiles and Hassall, 1898

### *Rhopalias* sp. 1

**Hosts:** *Biomphalaria straminea* and *Gundlachia ticaga* (Mollusca: Planorbidae)
**Locality:** Belo Horizonte, Minas Gerais, Brazil
**Prevalence:** 1/55 **(***B*. *straminea*) and 3/493 (*G*. *ticaga*)
**Deposited material:** UFMG-TRE 128 and UFMG-TRE 129

### Description

#### Cercariae (Figs 4A and 4B and 5A and 5B)

Body ovoid. Head collar without spines. Oral sucker spherical, subterminal. Prepharynx prominent, pharynx muscular, elongate. Ventral sucker spherical, post-equatorial, larger than oral sucker. Intestinal caeca absent. Cystogenous glands lateral along either side of body. Two or three large ovoid or spherical corpuscles (22–28 by 16–20) present inside each main duct of excretory system. Genital primordium, observed only in carmine-stained larvae, comprised of two masses of cells dorsal to ventral sucker. Excretory vesicle saccular, with a very short stem branching into two lateral arms extending anteriorly to oral sucker, with two to three spherical corpuscles (22–28 by 16–20) within each arm. Tail simple, assuming a figure-eight shape during swimming.

**Fig 4:** Cercaria of *Rhopalias* from *Biomphalaria straminea* from Brazil. (A) Whole view. (B) Detail of body. Cercariae from the same infected snail were genetically identified as *Rhopalias* sp. 1. Scale bars: 50 μm.

**Fig 5:** Larval stages of *Rhopalias* found in *Biomphalaria straminea* from Brazil. (A) Whole view of the cercaria stained with Nile blue sulphate. (B) Detail of the cercarial body stained with Nile blue sulphate. (C) Whole view of a redia. (D) Detail of the anterior region of a redia. (E) Metacercaria obtained experimentally in *Poecilia reticulata*. Cercariae from the same infected snail were molecularly identified as *Rhopalias* sp. 1. Scale bars: (A, B, D, E) 50 μm, (C) 100 μm.

#### Rediae (Fig 5C and 5D)

Body elongated. Pharynx subterminal. Caecum short. Several developed cercariae as well as developing cercariae and germ balls (not counted) present.

#### Metacercariae (Fig 5E)

Cyst ovoid to spherical, with thin, transparent cyst wall. Larvae with 2 to 3 large corpuscles inside each main excretory duct. Cyst obtained 24hrs after experimental infection of *P*. *reticulata* with cercariae measured 132 ± 7 (120–143) by 109 ± 3 (102–116).

### *Rhopalias* sp. 2

**Hosts:** Biomphalaria glabrata and Drepanotrema lucidum (Mollusca: Planorbidae);
Rhinella sp. (Amphibia: Bufonidae)
**Localities:** Januária and Patos de Minas, Minas Gerais, Brazil.
**Prevalence of infection:** 1/22 and 1/90 of B. glabrata and 8/8 of Rhinella sp. (Januária); 2/35 of D. lucidum (Patos de Minas).
**Deposited material:** UFMG-TRE 130 and UFMG-TRE 131

### Description

#### Cercariae (Fig 6A and 6B)

As in *Rhopalias* sp. 1.

**Fig 6:** Larval stages of *Rhopalias* found in *Biomphalaria glabrata* and *Rhinella* sp. from Brazil. (A) Whole view of a cercaria stained with Nile blue sulphate. (B) Detail of the body of a cercaria stained with neutral red. (C) Metacercariae found in a naturally infected tadpole. (D) Detail of a metacercaria. Cercariae from the same infected snail were genetically identified as *Rhopalias* sp. 2. Scale bars: (A, B, D) 50 μm, (C) 200 μm.

#### Probable metacercariae (Fig 6C and 6D)

Morphologically similar to that described for *Rhopalias* sp. 1. They measured 186 ± 4 (183–191) by 153 ± 31 (107–175). Despite the number and size of the excretory corpuscles being similar to those in cercariae, the conspecificity of the two stages requires further molecular study.

### *Rhopalias* sp. 3

**Host:** Drepanotrema lucidum
**Locality:** Dores do Indaiá
**Prevalence of infection:** 1/15.
**Deposited material:** not available.

### Description

**Cercariae.** As in Rhopalias sp. 1.

## Discussion

Although the parasitism of marsupials with *Rhopalias* spp. has been known since the early 19th century, the life cycles of digeneans in this genus remained unknown until now. In the present study, the occurrence of three species of *Rhopalias* in planorbid snails from Brazil was revealed by molecular data, representing the first identification of larval stages of species of this genus. The main distinctive characteristic present in cercariae of all three species of *Rhopalias* is the presence of few large granules in the main ducts of the excretory system, a trait that separates them from other known echinostomatid cercariae, which normally have small, numerous granules (e.g., *Drepanocephalus* spp., *Echinostoma* spp., *Echinoparyphium* spp., *Ribeiroia* spp.) [1]. The cercariae of *Rhopalias* spp. found in our study are morphologically indistinguishable from the larvae originally described as *Cercaria macrogranulosa* by Ruiz (1952) [33]. These cercariae were found in *B*. *glabrata* in the same locality (Belo Horizonte, Minas Gerais, Brazil) where our *Rhopalias* sp. 1 was found. Morphologically similar cercariae, also identified as *C*. *macrogranulosa*, were also reported in some species of planorbids from the genus *Biomphalaria* Preston, 1910 and *Drepanotrema* Crosse and Fischer, 1880 in Brazil (revised by Pinto and Melo [37]) and Argentina [36]. Likewise, *Cercaria echinostoma* 2 [34] and *Cercaria guaibensis* 8 [35], found in planorbids in southern Brazil, are also similar to cercariae described in the present study and thus, probably represent a species of *Rhopalias*, which requires further study for confirmation.

Our attempts at experimental infections using cercariae of *Rhopalias* sp. 1 failed to produce viable metacercariae. The contact of the cercariae with fish induced the encystment, suggesting that a cold-blooded aquatic vertebrate could act as the second intermediate host. Although *P*. *reticulata* appears not to be a susceptible host, the possibility of other fish species being infected in natural conditions cannot be ruled out. So far, the only experimental study involving larvae identified as *Cercaria macrogranulosa* was performed by Ostrowski of Núñez et al. (1990) [36] in Argentina, who reported the penetration and encystment of cercariae in tadpoles, revealing for the first time the possible involvement of amphibians in the transmission of the parasite. In the present study, metacercariae bearing 2–3 large refractile corpuscles in each main collecting duct of the excretory system were found in naturally infected tadpoles of *Rhinella* sp. collected in the same water body where *Rhopalias* sp. 2 was found in snails. This finding suggests that anurans play the role of the second intermediate host in the life cycles of *Rhopalias* spp. On the other hand, the absence of sequences for metacercariae from amphibians prevents us from confidently linking these metacercariae with *Rhopalias* sp. 2, even though they were found in the same habitat. Morphologically similar metacercariae were reported in the pharyngeal region of tadpoles of *Scinax nasicus* (Cope, 1862) and *Odontophrynus americanus* (Duméril and Bibron, 1841) in Argentina [38]. Similar to the previously published phylogeny [6], our phylogenetic analyses (Fig 1) placed *Rhopalias* spp. from Brazil and North America in a well-supported clade with species of *Ribeiroia* and *Cathaemasia*. It is important to note that anurans are also involved in the transmission of species from these two genera phylogenetically related to *Rhopalias* [6, 39–41]. Amphibians can be part of the diet of didelphid opossums [42–44], which enables the trophic transmission of *Rhopalias* spp. to the definitive host.

In this study, we attempted experimental infection aiming to obtain adult parasites using the probable metacercariae of *Rhopalias* sp. 2 found in naturally infected tadpoles. Despite the occasional reports of *Rhopalias* from non-marsupial hosts, including rodents [3], no adult worm was recovered in the mouse intestine. Similar experimental attempts were reported as successful with other echinostomatids, e. g., *Echinostoma* spp. [45–47]. New controlled studies are required to evaluate the susceptibility of rodents to *Rhopalias* spp., which could facilitate new experiments aiming at characterization of other aspects of host-parasite interrelationship involving these parasites (e.g., pathology, immunology, biochemistry).

The only available information on the life cycles of species of the genus *Rhopalias* is based on an unpublished thesis by Read [48], who obtained data on some aspects of the biology of *R*. *macracanthus* in North America. Read [48] was able to infect the physid snail *Physella gyrina* (Say, 1821) with eggs of *R*. *macracanthus* which resulted in the production of echinostome cercariae without a spined collar [48]. Those cercariae were significantly smaller (body: 100–145 by 56–65 μm; tail 70–200μm long) than the cercariae reported in the present study from Brazil. Importantly, the cercariae described by Read [48] are characterized by the presence of 10–15 small refractile granules (measuring 7 μm in diameter) in the main ducts of the excretory system. On the other hand, cercariae in Read [48] had visible caeca, unlike the larvae from Brazil. Read [48] successfully infected tadpoles as experimental second intermediate hosts and adult digeneans successfully developed in young opossums, but not in rats, guinea pigs, cat, and owls.

All cercarial samples obtained in our study were morphologically uniform and similar to previously described *C*. *macrogranulosa*. However, molecular data did not confirm the conspecificity among these cercariae. Although sequences of nuclear ribosomal DNA operon demonstrated lack of divergence among 5 out 6 samples from positive snails (the exception was the sample identified as *Rhopalias* sp. 3, with 0.1% divergence in 28S and 1.15% in ITS), data obtained for *nad*1 and *cox*1 unequivocally reveal the presence of different species of *Rhopalias* in our material. The larvae identified as *Rhopalias* sp. 2, were found in species from two different genera of planorbids (*Biomphalaria* and *Drepanotrema*) in two localities situated about 600 km apart. The divergence in *nad*1 gene between these isolates (2.1–2.4%) is similar to intraspecific divergence reported for other species of the Echinostomatidae [32, 49, 50]. In fact, higher interspecific divergences in *nad*1 were reported among species of *Echinostoma* (4.9–9.1%) [50, 51], *Patagifer* (6.76–8.55%) [49, 52], and *Drepanocephalus* (14.3%) [14]. On the other hand, samples of *Rhopalias* sp. 1 found in two phylogenetically distant genera of planorbids (*Biomphalaria* and *Gundlachia*) from the same locality were identical in *nad*1. Thus, our data indicate low specificity to planorbid first intermediate hosts can be verified in species of *Rhopalias*, at least for our *Rhopalias* sp. 1. Interestingly, two samples of *Rhopalias* sp. 2 collected from the same snail species (*B*. *glabrata*) and the same locality (Januária), but at different times, had differences in both *cox*1 (1.31%) and *nad*1 (1.83%) genes. Thus, further detailed studies are necessary to understand genetic diversity and population genetic structure of *Rhopalias* species found in this study.

Our results provide the first identification of planorbid snails as natural intermediate hosts of trematodes of the genus *Rhopalias*. Although physid snails were shown as potential experimental intermediate hosts of the North American *R*. *macracanthus* [48], this host-parasite association was not reported under natural conditions. Our discovery of snail intermediate hosts of species of *Rhopalias* using molecular tools came 7 decades after the first report of *Cercaria macrogranulosa* in Brazil. This can be due to the challenges in linking cercariae and adults of digeneans [9]. Therefore, the specific identification of the larvae reported herein requires obtaining DNA sequences from adult specimens of South American *Rhopalias* spp.

*Rhopalias coronatus* was the only *Rhopalias* species known in the state of Minas Gerais. It was found in the white-eared opossum, *Didelphis albiventris* Lund, 1840 from Belo Horizonte [53], the same area where cercariae of *Rhopalias* sp. 1 were found. Recently, *cox*1 sequences were obtained for Mexican isolates of *R*. *coronatus* [5], but that species is clearly distinct from our *Rhopalias* sp. 1 and *Rhopalias* sp. 2 (9.2–9.7% divergence in *cox*1). We cannot rule out the possibility of our *Rhopalias* sp. 3 being conspecific with one of the species sequenced in Mexico. Likewise, the larvae reported herein may belong to some of the other six species of *Rhopalias* known from marsupials in South America, namely *Rhopalias baculifer* Braun, 1900, *Rhopalias caballeroi* Kifune & Uyema, 1982, *Rhopalias caucensis* Rivillas, Caro, Carvajal & Vélez, 2004, *Rhopalias coronatus* (Rudolphi, 1819), *Rhopalias horridus* (Diesing, 1850) and *R*. *macracanthus* [8]. Of these, *R*. *baculifer*, *R*. *horridus* and *R*. *coronatus* were reported in Brazil [4, 7], and may correspond to some of the larvae reported herein.

Significant genetic differences between the sample of *R*. *macracanthus* from the USA sequenced in the present study and sequences of the same species from Mexico [5] indicate the possibility of these isolates belonging to different species of *Rhopalias*. It should be noted that the authors pointed out some morphological differences in proboscis spines between their specimens from Mexico and the original description [5]. Considering that *R*. *macracanthus* was originally described from the Virginia opossum in the USA [4], it is more likely that our isolate from the USA corresponds to this species. Additional sequencing and detailed morphological studies of specimens from both Mexico and the USA, including hologenophores, are necessary to answer this question.

Similar to observations in some other groups of digeneans, our results demonstrated that despite the usefulness of the nuclear ribosomal RNA sequences for phylogenetic inference at levels of genera and higher taxa, their level of variation can be too low for the specific level. This fact was verified between our *Rhopalias* sp. 1 and *Rhopalias* sp. 2. In a study carried out in Mexico, *cox*1 sequences (barcoding region) were obtained for three species of *Rhopalias* [5]. In our study, we successfully amplified the same region of *cox*1 only from one of our samples (*Rhopalias* sp. 1) using the primers Dice-1 and Dice-11 developed by Van Steenkiste et al. [27]. Instead, we successfully amplified and sequenced *Rhopalias* sp. 2 using the combination of Dice-1 and BarCox-R primers. Unlike *cox*1, partial sequences of the fragment of the *nad*1 gene have been widely used in studies of the Echinostomatoidea [12–17;49–52]. Amplification and sequencing of this fragment in our study of *Rhopalias* spp. was not problematic; therefore, its use is encouraged in future studies involving these digeneans.

More than 30 species of digeneans, including six species of *Rhopalias*, have been reported in South American marsupials thus far [8]; remarkably, none of these species had molecular data available prior to our study. This deficiency in the generation of molecular data is particularly obvious in South America [54]. Thus, obtaining sequence data from quality, well-fixed and identified adult specimens of *Rhopalias* spp. is critical for future progress in our knowledge of the biology and taxonomy of digeneans parasitic in marsupials.

## Supporting information

S1 Table Information on sequences of representative species of the superfamily Echinostomatoidea used in the phylogenetic analyses. (XLSX)

## References

[1] YamagutiS. Synopsis of Digenetic Trematodes of Vertebrates. vol. 1. Keigaku Publishing Company: Tokyo; 1971.

[2] MarshallME, MillerGC. Some digenetic trematodes from Ecuadorian bats including five new species and one new genus. J. Parasitol. 1979;65: 909–917.

[3] RadevV, GardnerSL, KanevI. Family Rhopaliidae Looss, 1899. In: Keys to the Trematoda, JonesA, BrayRA, and GibsonDI (eds). London, U.K.: CAB International and The Natural History Museum; 2005. p. 119–120.

[4] HaverkostTR, GardnerSL. A review of species in the genus *Rhopalias* (Rudolphi, 1819). J. Parasitol. 2008;94: 716–726.1860580110.1645/GE-1423.1

[5] López-CaballeroJ, Mata-LópezR, Pérez Ponce de LeónG. Molecular data reveal a new species of *Rhopalias* Stiles & Hassall, 1898 (Digenea, Echinostomatidae) in the Common opossum, *Didelphis marsupialis* L. (Mammalia, Didelphidae) in the Yucatán Peninsula, Mexico. ZooKeys 2019;854: 145.3123982110.3897/zookeys.854.34549PMC6580842

[6] TkachVV, KudlaiO, KostadinovaA. Molecular phylogeny and systematics of the Echinostomatoidea Looss, 1899 (Platyhelminthes: Digenea). Int. J. Parasitol. 2016;46: 171–185. doi: 10.1016/j.ijpara.2015.11.001 26699402

[7] GomesDC, VicenteJJ. Estudo do gênero *Rhopalias* Stiles & Hassall, 1898 (Trematoda, Rhopaliasidae). Mem. Inst. Oswaldo Cruz 1972; 70:115–133.

[8] FernandesBMM, JustoCN, CárdenasMQ, CohenSC. South American trematodes parasites of birds and mammals. Rio de Janeiro: FIOCRUZ; 2015.

[9] Blasco-CostaI, PoulinR. Parasite life-cycle studies: a plea to resurrect an old parasitological tradition. J. Helminthol. 2017;91: 647–656. doi: 10.1017/S0022149X16000924 28166844

[10] Blasco-CostaI, PoulinR, PresswellB. Species of *Apatemon* Szidat, 1928 and *Australapatemon* Sudarikov, 1959 (Trematoda: Strigeidae) from New Zealand: linking and characterising life cycle stages with morphology and molecules. Par. Res. 2016;115: 271–289.10.1007/s00436-015-4744-026385467

[11] Blasco-CostaI, LockeSA. Life history, systematics, and evolution of the Diplostomoidea Poirier, 1886: progress, promises and challenges emerging from molecular studies. Adv. Parasitol. 2017;98: 167–225. doi: 10.1016/bs.apar.2017.05.001 28942769

[12] PrasadPK, GoswamiL, TandonV, ChatterjeeA. PCR-based molecular characterization and in silico analysis of food-borne trematode parasites Paragonimus westermani, Fasciolopsis buski and Fasciola gigantica from Northeast India using ITS2 rDNA. Bioinformation 2011;6: 64–68. doi: 10.6026/97320630006064 21544167PMC3082855

[13] Sereno-UribeAL, Pinacho-PinachoCD, CorderoVS, García-VarelaM. Morphological and molecular analyses of larval and adult stages of Echinoparyphium recurvatum von Linstow 1873 (Digenea: Echinostomatidae) from central Mexico. J. Helminthol. 2014; 89: 458–464. doi: 10.1017/S0022149X14000297 24739119

[14] PintoHA, GriffinMJ, QuiniouSM, WareC, MeloAL. Biomphalaria straminea (Mollusca: Planorbidae) as an intermediate host of Drepanocephalus spp. (Trematoda: Echinostomatidae) in Brazil: a morphological and molecular study. Par. Res. 2016;115: 51–62.10.1007/s00436-015-4469-025982569

[15] CechG, MolnárK, SzékelyC. Molecular biological studies of adult and metacercarial stages of Petasiger exaeretus Dietz, 1909 (Digenea: Echinostomatidae). Acta Vet. Hung. 2017;65: 198–207. doi: 10.1556/004.2017.020 28605968

[16] AssisJCA, López-HernándezD, FavorettoS, MeloAL, MartinsNRS, PintoHA. Identification of a transmission focus of the avian tracheal trematode Typhlocoelum cucumerinum (Trematoda: Cyclocoelidae): diagnosis, life cycle and molecular phylogeny. Parasitology 2021;148: 1383–1391.3410310710.1017/S0031182021000986PMC11010135

[17] GalaktionovKV, SolovyevaAI, MiroliubovA. Elucidation of Himasthla leptosoma (Creplin, 1829) Dietz, 1909 (Digenea, Himasthlidae) life cycle with insights into species composition of the north Atlantic Himasthla associated with periwinkles Littorina spp. Par. Res. 2021;120: 1649–1668. doi: 10.1007/s00436-021-07117-8 33712931

[18] Pérez-Ponce de LeónG, Hernández-MenaDI. Testing the higher-level phylogenetic classification of Digenea (Platyhelminthes, Trematoda) based on nuclear rDNA sequences before entering the age of the ‘next-generation’ Tree of Life. J. Helminthol. 2019;93: 260–276. doi: 10.1017/S0022149X19000191 30973318

[19] ParaenseWL. Estado atual da sistemática dos planorbídeos brasileiros. Arq. Mus. Nac. 1975;55: 105–128.

[20] SantosSB. Estado atual do conhecimento dos ancilídeos na América do Sul (Mollusca: Gastropoda: Pulmonata: Basommatophora). Rev. Biol. Trop. 2003; 191–224.

[21] SimoneLRL, BuniotoTC, AvelarWE, HayashiC. Morphology and biological aspects of Gundlachia ticaga from SE Brazil (Gastropoda: Basommatophora: Ancylidae). Arch. Molluskenkd. 2012;141: 21–30.

[22] LacerdaL, LacerdaLE, MiyahiraI. First record and range extension of the freshwater limpet Gundlachia radiata (Guilding, 1828) (Mollusca: Gastropoda: Planorbidae) from southeast Brazil. Check List 2013;9: 125–128.

[23] TkachVV, LittlewoodDT, OlsonPD, KinsellaJM, SwiderskiZ. Molecular phylogenetic analysis of the Microphalloidea Ward, 1901 (Trematoda: Digenea). Syst. Parasitol. 2003;56: 1–15. doi: 10.1023/a:1025546001611 12975618

[24] LutonK, WalkerD, BlairD. Comparisons of ribosomal internal transcribed spacers from two congeneric species of flukes (Platyhelminthes: Trematoda: Digenea). Mol. Biochem. Parasitol. 1992;56: 323–328. doi: 10.1016/0166-6851(92)90181-i 1484553

[25] KostadinovaA, HerniouEA, BarrettJ, LittlewoodDTJ. Phylogenetic relationships of Echinostoma Rudolphi, 1809 (Digenea: Echinostomatidae) and related genera re-assessed via DNA and morphological analyses. Syst. Parasitol. 2003;54: 159–176. doi: 10.1023/a:1022681123340 12652069

[26] BowlesJ, McManusDP. NADH dehydrogenase 1 gene sequences compared for species and strains of the genus *Echinococcus*. Int. J. Parasitol. 1993;23: 969–972.810619110.1016/0020-7519(93)90065-7

[27] Van SteenkisteN, LockeSA, CastelinM, MarcoglieseDJ, AbbottCL. New primers for DNA barcoding of digeneans and cestodes (Platyhelminthes). Mol. Ecol. Resour. 2015;15: 945–952. doi: 10.1111/1755-0998.12358 25490869

[28] PaithankarKR, PrasadKS. Precipitation of DNA by polyethylene glycol and ethanol. Nucleic Acids Res. 1991;19: 1346. doi: 10.1093/nar/19.6.1346 2030954PMC333871

[29] KumarS, StecherG, LiM, KnyazC, TamuraK. MEGA X: molecular evolutionary genetics analysis across computing platforms. Mol. Biol. Evol. 2018;35: 1547–1549. doi: 10.1093/molbev/msy096 29722887PMC5967553

[30] DereeperA, GuignonV, BlancG, AudicS, BuffetS, ChevenetF, et al. Phylogeny.fr: robust phylogenetic analysis for the non-specialist. Nucleic Acids Res. 2008; 36: W465–W469. doi: 10.1093/nar/gkn180 18424797PMC2447785

[31] RonquistF, TeslenkoM, van der MarkP, AyresDL, DarlingA, HöhnaS, et al. Software for systematics and evolution MrBayers 3.2: efficient bayesian phylogenetic inference and model choice across a large model space. Syst. Biol. 2012;61: 539–542.2235772710.1093/sysbio/sys029PMC3329765

[32] Rambaut A, Drummond AJ. FigTree. 2012; Available from http://tree.bio.ed.ac.uk/software/figtree/. Accessed Apr 2020.

[33] RuizJM. Contribuição ao estudo das formas larvares de trematódeos brasileiros. 3. Fauna de Belo Horizonte e Jaboticatubas, Estado de Minas Gerais. Mem. Inst. Butantan 1952;24: 45–62.13012831

[34] Veitenheimer-MendesIL. Cercárias em moluscos planorbídeos de Camaquã, Rio Grande do Sul, Brasil. Rev. Bras. Biol. 1982;42: 545–551.

[35] Veitenheimer-MendesIL, OhlweilerFP, BlumC. Gastrópodes límnicos (Mollusca), hospedeiros intermediários de trematódeos (Platyhelminthes) em Porto Alegre e Viamão, Rio Grande do Sul. Biociências 1995;3: 73–84.

[36] Ostrowski de NúñezM, HamannMI, RumiA. Larval trematodes of Schistosoma mansoni transmiting snail: Biomphalaria spp. in northeastern Argentina. Acta Parasitol. Pol. 1990;35: 85–96.

[37] PintoHA, MeloAL. A checklist of cercariae (Trematoda: Digenea) in molluscs from Brazil. Zootaxa. 2013;3666: 449–475. doi: 10.11646/zootaxa.3666.4.3 26217863

[38] HamannMI, GonzálezCE. Larval digenetic trematodes in tadpoles of six amphibian species from northeastern Argentina. J. Parasitol. 2009;95: 623–628. doi: 10.1645/GE-1738.1 19045934

[39] SzidatL. Beitrage zum Aufbau eines naturlichen systems der Trematoden. I. Die entwicklung von Echinocercaria choanophila U. Szidat zu Cathaemasia hians und die Ableitung der Fasciolidae von den Echinostomatidae. Z. Parasitenkd. 1939;11: 239–283.

[40] YamagutiSA. Synoptical Review of Life Histories of Digenetic Trematodes of Vertebrates with Special Reference to the Morphology of their Larval Forms. Keigaku Publishing Co.: Tokyo; 1975.

[41] JohnsonPTJ, SutherlandDR, KinsellaJM, LundeKB. Review of the trematode genus Ribeiroia (Psilostomidae): ecology, life history and pathogenesis with special emphasis on the amphibian malformation problem. Adv. Parasitol. 2004;57: 191–253. doi: 10.1016/S0065-308X(04)57003-3 15504539

[42] StiegltizWO, KlimstraWD. Dietary pattern of the Virginia opossum, Didelphis virginianus Kerr, late summer-winter, southern Illinois. Trans. Ill. State Acad. Sci.1962; 55: 198–208.

[43] ValerioCE. A gran capacidad adaptiva del zorro pelon (Didelphis masrupialis Linn). Rev. Univ. Costa Rica 1969;26: 43–44.

[44] ToledoLF, RibeiroRS, HaddadCFB. Anurans as prey: an exploratory analysis and size relationships between predators and their prey. J. Zool. 2007; 271: 170–177.

[45] McMasterRP, HuffmanJE, FriedB. The effect of dexamethasone on the course of Echinostoma caproni and E. trivolvis infections in the golden hamster (Mesocricetus auratus). Par. Res. 1995;81: 518–521. doi: 10.1007/BF00931795 7567911

[46] FujinoT, IchikawaH, FriedB, FukudaK. The expulsion of Echinostoma trivolvis: suppressive effects of dexamethasone on goblet cell hyperplasia and worm rejection in C3H/HeN mice. Parasite. 1996;3: 283–289. doi: 10.1051/parasite/1996033283 9008738

[47] FriedB, MuellerTJ, FrazerBA. Observations on *Echinostoma revolutum* and *Echinostoma trivolvis* in single and concurrent infections in domestic chicks. Int. J. Parasitol. 1997;27: 1319–1322.942171810.1016/s0020-7519(97)00100-8

[48] Read CP. The life history and morphology of Rhopalias macracanthus Chandler (Trematoda) [dissertation]. Houston, Texas: William Marsh Rice Institute 1948.

[49] LaidemittMR, BrantSV, MutukuMW, MkojiGM, LokerES. The diverse echinostomes from East Africa: with a focus on species that use *Biomphalaria* and *Bulinus* as intermediate hosts. Acta Trop. 2019;193: 38–49.3071053110.1016/j.actatropica.2019.01.025PMC6461134

[50] GeorgievaS, SelbachC, FaltýnkováA, SoldánováM, SuresB, SkírnissonK, et al. New cryptic species of the ‘revolutum’ group of Echinostoma (Digenea: Echinostomatidae) revealed by molecular and morphological data. Parasites Vectors. 2013;6: 64. doi: 10.1186/1756-3305-6-64 23497579PMC3605289

[51] MohantaUK, WatanabeT, OhariY, ItagakiT. Characterization of *Echinostoma revolutum* and *Echinostoma robustum* from ducks in Bangladesh based on morphology, nuclear ribosomal ITS2 and mitochondrial nad1 sequences. Parasitol. Int. 2019;69: 1–7.3044519910.1016/j.parint.2018.11.002

[52] Sereno-UribeAL, González-GarcíaMT, Ortega-OlivaresMP, López-JiménezA, García-VarelaM, Andrade-GómezL. First record of Patagifer bilobus (Rudolphi, 1819) Dietz, 1909 (Digenea: Echinostomatidae), with a morphological and molecular characterization from two threskiornithid species in Mexico. Parasitol. Res. 2022;121: 1921–1935. doi: 10.1007/s00436-022-07526-3 35488923

[53] Quintão e SilvaM, CostaHM. Helminths of white-bellied opossum from Brazil. J. Wildl. Dis. 1999;35: 371–374. doi: 10.7589/0090-3558-35.2.371 10231765

[54] PoulinR, JorgeF. The geography of parasite discovery across taxa and over time. Parasitology. 2019;146: 168–175. doi: 10.1017/S003118201800118X 30012225

